The article "Sorting machineries: how platelet-dense granules differ from α-granules" was published in 2018. Journal: Biosci Rep.

# Sorting machineries: how platelet-dense granules differ from α-granules

**DOI:** 10.1042/BSR20180458

**Published:** 2018-09-07

**Authors:** Yuanying Chen, Yefeng Yuan, Wei Li

**Affiliations:** Beijing Key Laboratory for Genetics of Birth Defects, MOE Key Laboratory of Major Diseases in Children, Center for Medical Genetics, Beijing Pediatric Research Institute, Beijing Children’s Hospital, Capital Medical University, National Center for Children’s Health, Beijing, China

**Keywords:** inherited platelet disorders, organelle biogenesis, platelet granules, sorting machineries

## Abstract

Platelets respond to vascular injury via surface receptor stimulation and signaling events to trigger aggregation, procoagulant activation, and granule secretion during hemostasis, thrombosis, and vascular remodeling. Platelets contain three major types of secretory granules including dense granules (or δ-granules, DGs), α-granules (AGs), and lysosomes. The contents of platelet granules are specific. Platelet DGs store polyphosphate and small molecules such as ADP, ATP, Ca^2+^, and serotonin, while AGs package most of the proteins that platelets release. The platelet DGs and AGs are regarded as being budded from the endosomes and the *trans*-Golgi network (TGN), respectively, and then matured from multivesicular bodies (MVBs). However, the sorting machineries between DGs and AGs are different. Inherited platelet disorders are associated with deficiency of DGs and AGs, leading to bleeding diathesis in patients with Hermansky–Pudlak syndrome (HPS), gray platelet syndrome (GPS), and arthrogryposis, renal dysfunction, and cholestasis syndrome (ARC). Here, we reviewed the current understanding about how DGs differ from AGs in structure, biogenesis, and function. In particular, we focus on the sorting machineries that are involved in the formation of these two types of granules to provide insights into their diverse biological functions.

## Introduction

Platelets are small and anucleate blood cells, which originated from bone marrow megakaryocytes (MKs). The fundamental function of circulating platelets is to form aggregates that are adhered to the injured vessel wall to prevent bleeding [1]. Platelet granule exocytosis is critical to platelet function and participates in platelet activities [2]. Platelets contain three types of well-known secretory granules including dense granules (or δ-granules, DGs), α-granules (AGs), lysosomes, and a recently described type T granule, which is defined by the presence of toll-like receptor (TLR9) and protein disulphide isomerase (PDI) during pro-platelet production [3–5]. Platelet activation is mediated by secreted molecules, which are stored in DGs and AGs. These two granules carry distinct cargos and vary in biogenesis and function. Most of the proteins that platelets release from AGs are coagulation factors, adhesive molecules, growth factors, angiogenic and immune mediators [6]. In comparison with AGs that package hundreds of proteins, DGs contain relatively few types of small molecules including serotonin, ADP, ATP, Ca^2+^, Mg^2+^, K^+^, pyrophosphate, and polyphosphate [7]. Platelets that respond to low-level agonists such as collagen or thrombin are promoted by autocrine and paracrine pathways due to the secretion of ADP and ATP from DGs [8].

Previous studies have shown that deficiency or absence of AGs is associated with two inherited platelet disorders: gray platelet syndrome (GPS) and arthrogryposis, renal dysfunction, and cholestasis syndrome (ARC). Further studies revealed that platelets from GPS patients have loss-of-function mutations in *NBEAL2*, while platelets from ARC patients have loss-of-function mutations in vacuolar protein sorting 33 homolog B (*VPS33B*) or *VPS16B*. These studies suggest that *NBEAL2, VPS33B*, and *VPS16B* are involved in AG biogenesis and function [9–11]. DG is a type of lysosome-related organelle (LRO) [12]. The bleeding diathesis in patients with Hermansky–Pudlak syndrome (HPS) or Chediak–Higashi syndrome (CHS) is caused by DG deficiency [12–14]. HPS is characterized by oculocutaneous albinism (OCA), bleeding tendency, and ceroid deposition which lead to lung fibrosis, colitis, and cardiomyopathy. CHS is characterized by variable degrees of OCA, easy bleeding, and recurrent infections [12]. HPS and CHS are syndromic albinism caused by mutations in genes such as *HPS1–10* and *CHS1*, respectively, which encode proteins HPS1, adaptor protein (AP-3) β3A, HPS3, HPS4, HPS5, HPS6, Dysbindin, BLOS3, Pallidin, AP-3 δ, and LYST [12,15]. These proteins form complexes such as biogenesis of LRO complex (BLOC)-1/-2/-3, AP-3 which are involved in endolysosomal trafficking [12]. The underlying mechanism of DG biogenesis is relatively lacking and has been assumed to be similar with other LRO such as melanosome that is defective in HPS and CHS [16,17]. Several protein complexes such as the BLOCs, homotypic fusion and vacuole protein sorting complex (HOPS), and class C core vacuole/endosome tethering complex (CORVET) are involved in DG biogenesis [7]. Based on the current knowledge, this review will provide an overview on the structures, biogenesis, and biological functions of DGs and AGs to understand how platelet DGs differ from AGs at the angle of sorting machineries.

## Structures of AGs and DGs

### AG structure

The initial findings about AG structure were based on thin section EM. In normal circulating platelets, AGs are the most abundant platelet granules, numbering approximately 50–80 per cell [18]. AGs are relatively large with 200–500 nm in diameter and constitute approximately 10% of the platelet volume [19]. Based on EM, proteomics, platelet activation studies, and super resolution fluorescence microscopy, the structure and protein organization of AGs have been depicted. Briefly, the morphology of AG is round or ovoid and it contains an electron-dense nucleoid, lumenal matrix, and a peripheral cluster of tubules [20]. AGs have hundreds of proteins including typically membrane-associated receptors P-selectin, soluble fibrinogen (FGN), and secretory von Willebrand factor (vWF) [6]. Recently, 3D structured illumination microscopy (3D-SIM) and direct stochastical optical reconstruction microscopy (dSTORM) have been applied to measure the differential distribution of FGN and vWF. These techniques show that VWF and FGN overlap in a small portion (approximately 18%) [21,22]. Different classes of AGs have been characterized. One class is the spherical granules exhibiting a heterogeneous matrix substructure with electron-dense and electron-lucent zones, containing 12-nm vWF tubules. The second class is the multivesicular subtype displaying a multitude of free luminal membrane vesicles. The third class is a distinct population of approximately 50 nm wide tubular granules, which have been designated tubular AGs [23]. These findings suggest that AG may have different populations containing different cargos. However, the underlying mechanisms for the biogenesis of these classes are unknown. It will be interesting to explore whether different sorting machineries are involved in the formation of these AG subtypes.

### Dense granule structure

In comparison with the number of AGs in platelets, DGs are much less. Normally, each human platelet contains only three to eight DGs with 200–300 nm in diameter [7]. DGs, with a luminal pH of 6.1, belong to a family of LRO which are acidic compartments [16,24]. Unlike AGs with hundreds of proteins, DGs contain serotonin, calcium, pyrophosphate, and a non-metabolic adenine nucleotide pool of ADP and ATP that play pivotal role in platelet activation. During exocytosis, both ADP and serotonin act as platelet agonists and are important to activate circulating platelets to be recruited to the site of injury. Calcium enables DG an electron-dense property and allows them to be viewed by EM without additional staining [24]. Although fluorescence microscopy and super-resolution fluorescence microscopy have been used to observe DGs, EM remains to be the best method to quantitate the number of DGs [7,25,26]. DGs are easily detected in unfixed, unstained whole-mount preparations, and also in thin sections of properly fixed platelets using TEM [27]. Using the whole mount technique, DGs are inherently opaque and can be quantitated under the fields. Thus, as for DG number counting, the whole mount EM method has become a standard procedure to determine the presence or absence of DGs in diagnosing patients with HPS or CHS. When fixing in thin sections of platelets and MKs and treated with osmic acid, DGs can be clearly visualized as membrane-bound structures with dense cores by EM [27]. For super-resolution microscopy, it is less expensive and less labor intensive than using EM. This could have potential application in diagnosing patients with storage pool deficiency (SPD) of either AG or DG [25].

## Biogenesis of AGs and DGs

Platelets are derived from MKs through the extending cytoplasmic proplatelets via processes involving microtubules and dynein [28]. During platelet formation, granules are generated by packaging proteins to exert physiological functions. These proteins are sorted into the granules by a number of sorting machineries during granule biogenesis.

### AG biogenesis

AG development involves trafficking and sorting of proteins mediated by vesicles that bud from the membranes of one cellular compartment and fuse with another compartment [6]. Using ultrathin cryosectioning and immunogold cytochemistry to study AG in MKs and platelets, it has been suggested that the precursors of AGs bud from either the *trans*-Golgi network (TGN) or the plasma membrane and then are directed to multivesicular bodies (MVBs)/late endosomes (LEs) [29]. In MKs, two types of MVBs have been described in the process of AG biogenesis. Both newly synthesized cargos from TGN or endocytosed proteins from plasma membrane are transported into immature MVB type I (MVB I) characterized by the presence of internal vesicles via early endosomes. MVB I matures to MVB type II (MVB II) which contains both internal vesicles and an electron-dense matrix, and subsequently matures to AG (Figure 1).

**Figure 1:** A model for the biogenesis of platelet AGs and DGs In MKs, some integral or soluble cargos of AGs and DGs are endocytosed into early endosomes. In the process of AG biogenesis, both newly synthesized cargos from TGN and endocytosed proteins from the plasma membrane are transported into MVB I or MVB II. During the maturation of AGs, *VPS33B, VPS16B*, and *NBEAL2* proteins play pivotal roles. MVBs are also involved in the formation of DGs. DG cargos are sorted by AP-3 complex at the endosomal tubules, which is likely stabilized by BLOC-1. AP-3 binds the sorting signals present in the cytosolic tails of cargo proteins. The functions of BLOC-2 and BLOC-3 in DG biogenesis are less understood. They are suspected to act downstream of BLOC-1 and AP-3. BLOC-2 interacts physically with BLOC-1 as well as with Rab38/Rab32. Rab38/Rab32 act in trafficking of cargos from early/recycling endosomes to mature DGs in MKs, and colocalize with AP-3 and clathrin-labeled structures and DGs. BLOC-3 acts as a guanine nucleotide exchange factor specifically for Rab32 and Rab38 and thus pinpoint BLOC-3 to DG biogenesis.

The study of molecular pathogenesis underlying GPS and ARC syndrome provides insights into AG biogenesis. Mutations in *VPS33B*, a novel Sec1/Munc18 protein, lead to ARC syndrome [10]. In wild-type human MKs, VPS33B colocalized mostly with AGs and moderately with late endosomes. Patients with *VPS33B* mutations detected no VPS33B protein expression in their fibroblasts by immunoblotting. Consequently, platelet AGs were completely absent from ARC syndrome platelets. In addition, soluble AG cargos including platelet factor 4 (PF4), vWF, β-thromboglobulin, thrombospondin 1, endocytosed FGN, and membrane-bound P-selectin could not be detected in platelets [10]. These observations indicate that VPS33B is required for the production of AGs at an early stage when MVB II are formed. Recently, VPS16B was identified as a VPS33B-binding protein that is also required for AG biogenesis [11]. ARC syndrome with *VPS16B* mutation revealed a complete loss of AGs. Soluble and membrane-bound AG proteins were reduced or undetectable, suggesting that both releasable and membrane-bound AG constituents were absent. Stable expression of GFP-VPS16B in Dami cells showed that VPS16B colocalized with AGs, late endosomes, and TGN, indicating that VPS16B, together with its binding partner VPS33B, is essential for AG biogenesis in MKs and platelets [11].

The function of VPS33B in AG trafficking has been confirmed in a mouse model [30]. By generating a tamoxifen-inducible mouse model of VPS33B deficiency, *Vps33b^fl/fl^-ER^T2^*, the authors found a marked reduction in AG counts and the presence of small granule-like structures in platelets by phenocopying the platelet phenotypes in ARC patients. Analysis of bone marrow-derived MKs from *Vps33b^fl/fl^-ER^T2^* mice revealed a reduction in mature MVB II and an accumulation of large vacuoles, which may result from mis-sorting of proteins during trafficking. Very less cargo protein such as vWF was transported from MVB I to MVB II [30], suggesting that VPS33B in complex with VPS16B plays an essential role in trafficking cargo proteins thus affects AG biogenesis and formation.

Genetic analyses have shown that mutations in *NBEAL2*, which encodes neurobeachin-like 2 protein, lead to GPS [9]. GPS platelets had reduced proteins in AGs and the MK-synthesized cargo proteins were absent, while the levels of endocytosed proteins such as FGN were less affected [31,32]. Immuno-gold EM studies showed that P-selectin-positive membranes were vacuole-like and matrix-deficient vesicles [33]. With immuno-EM and fluorescence microscopy, the authors observed that in MKs from GPS patients and *Nbeal2^−/−^* mice, vWF initially appeared within small vesicles near the Golgi that failed to mature into AGs and were released into the demarcation membrane system (DMS, a major element of the MK cytoplasmic maturation process [34]) instead, abnormally distributing vWF onto the outer cell surface [35,36]. In *Nbeal2^−/−^* mice, MK morphology and maturation were defective in decreased ploidy and proplatelet formation [36]. It is suggested that GPS with *NBEAL2* mutations has a deficiency in cargo protein sorting into AGs.

Although VPS33B, VPS16B, and NEBAL2 are implicated in AG biogenesis, the detail mechanisms of how they regulate AG biogenesis remain poorly understood. It has been suggested that both VPS33B and VPS16B are involved in protein sorting and trafficking, which is required for delivery of endocytosed cargos to lysosomes. The VPS33B–VPS16B complex is essential for late endosome-lysosome fusion and endosomal recycling [37]. VPS33B–VPS16B complex interacts with the active form of Rab11a, which is involved in apical membrane protein sorting. From liver samples of individuals with ARC, abnormal expression of E-cadherin, and the apical membrane protein CEACAM5 were found, suggesting the role of VPS33B–VPS16B complex in protein sorting and trafficking [38]. VPS16B has also been reported to interact with lysyl hydroxylase 3 (LH3) and to regulate its sorting into post-Golgi collagen carriers [39]. But the molecular mechanisms of VPS33B-VPS16B complex in regulating AG biogenesis remain to be elucidated.

### Dense granule biogenesis

DGs, as a member of LRO [16,17], share several features of LRO including an acidic lumen and possible biogenesis machineries [7]. The biogenesis of DGs has been assumed to have similar mechanisms as other LRO such as melanosome, which involves a specialized biogenesis mechanism that connects the secretory and endocytic pathways (Figure 1). Due to the difficulty in manipulating granule biogenesis experiments in MKs, the DG biogenesis mechanisms are poorly understood [5,40]. However, some progress has been made using isolated primary MKs to provide insights into the protein sorting machineries during platelet DG biogenesis. In general, different from AG biogenesis, DGs originate directly from endosomes, not from the TGN. Although MVBs are likely the precursors of DGs, AGs, and lysosomes, the evolving processes from MVBs to these three types of organelles require different protein sorting and regulating machineries. After originated from MVBs, DG maturation acquires newly synthesized DG proteins through sorting machineries and intermediate compartments of the endosomal transport (Figure 1) [7,41].

The AP-3 complex was originally identified by its homology with the clathrin-associated AP complexes AP-1 and AP-2, which are involved in vesicle trafficking [42,43]. AP-3 mediates transport of integral membrane proteins from tubular domains of early/recycling endosomes to lysosomes and LROs [44,45]. The function of AP-3 in the biogenesis of DGs and LROs is demonstrated by mutations of AP-3 in HPS mouse models, pearl and mocha, also in HPS-2 and HPS-10 patients [46–48]. AP-3 recognizes dileucine- and tyrosine-based sorting signals in the cytosolic tail of integral membrane protein cargos and packages them into transporting vesicles destined for LRO [7,45,49]. Based on the characteristics of AP-3 protein, several candidate DG integral membrane protein components have the cytosolic tails harboring sequences of consensus dileucine- and tyrosine-based sorting signals [7]. For example, the protein SLC35D3, a member of the nucleotide sugar transporter family, is required for platelet DG biogenesis and its mutation causes DG deficiency in mice [50,51]. Immunofluorescence showed that SLC35D3 populates early endosomal tubules labeled with syntaxin 13 and transferrin receptor in MKs. In AP-3 deficient mice platelets, SLC35D3 was decreased, suggesting that AP-3 likely regulates SLC35D3 trafficking to DGs during its biogenesis [51]. Other candidate AP-3 cargo proteins are LAMP2 and the serotonin transporter vesicular monoamine transporter 2 (VMAT2) located on the DG membrane. The mutation forms of dileucine- and tyrosine-based sorting signals of LAMP2 and VMAT2 were mislocalized to the plasma membrane [49]. These observations suggest that AP-3 and the sorting signals of cargo proteins mediate transport of newly synthesized integral membrane proteins from endosomes to DGs.

Other machineries in regulating DG biogenesis by sorting cargos from endosomes are the BLOC complexes including BLOC-1, BLOC-2, and BLOC-3. BLOC-1 is a heteromeric complex composed of eight subunits: BLOS1 (BLOC1S1), BLOS2 (BLOC1S2), BLOS3 (BLOC1S3), Cappuccino (BLOS4 or BLOC1S4), Muted (BLOS5 or BLOC1S5), Pallidin (BLOS6 or BLOC1S6), Snapin (BLOS7 or BLOC1S7), and Dysbindin (BLOC1S8 or DTNBP1) [12,52,53]. BLOC-2 is composed of HPS3, HPS5, and HPS6 proteins [54]. BLOC-3 is composed of HPS1 and HPS4 [55]. The mutations of most genes encoding proteins of BLOC subunits have been found in HPS patients or mice. The mechanisms of BLOCs in regulating DG biogenesis are very limited, but the functions of BLOCs in delivering integral membrane proteins to maturing melanosomes are quite clear which may be inferred in DG biogenesis. For instance, BLOC-1 interacts physically with AP-3 and the endosomal syntaxin 13. It is likely that BLOC-1 performs similar functions in transporting DG proteins during organelle biogenesis [56]. Other evidence supported this idea that SLC35D3 steady-state levels in platelets from BLOC-1 deficient mice were decreased as was also observed in AP-3 deficient mice [51]. Furthermore, BLOC-2 interacts physically with BLOC-1 as well as with Rab38 and Rab32, two small GTPases that function in DG biogenesis [49,56]. Rab32 and Rab38 act in trafficking of cargos from early/recycling endosomes to mature DGs in MKs, and colocalizes with AP-3 and clathrin-labeled structures and DGs [49,57]. The function of BLOC-3 in DG biogenesis is less understood. Platelets from an HPS4 patient showed reduced MRP4 staining, the nucleotide transporter which is highly expressed in DGs, and MRP4 was mostly found on the plasma membrane. The mislocation of MRP4 suggests that BLOC-3 may function in transport of MRP4 to DGs [58]. Recombinant BLOC-3 has guanine nucleotide exchange factor (GEF) activity specially for Rab32 and Rab38 and thus pinpoint BLOC-3 to the trafficking machinery that transports cargos to DGs (Figure 1) [59].

Other factor that may be involved in platelet dense granule biogenesis is VPS33A, a subunit of HOPS complex [60]. HOPS complex is composed of six subunits: VPS33A, VPS11, VPS16, VPS18, VPS39, and VPS41. Four subunits of HOPS (VPS33A, VPS11, VPS16, and VPS18) are shared with a related complex known as CORVET [61]. HOPS and CORVET function as tethering complexes in membrane trafficking and facilitate SNARE-mediated membrane fusion. It is reported that VPS33A regulates the formation of cognate SNARE complexes in driving membrane fusion [62] which may extend their function in generating the precursor MVB compartment and/or mediating tethering and fusion of DG cargo-containing vesicles with MVBs [7]. Notably, VPS33B, which functions in AG biogenesis, is related to VPS33A. Thus, VPS33A and VPS33B diverse the sorting routes in DG and AG biogenesis.

DG contains serotonin, calcium, pyrophosphate, and a non-metabolic adenine nucleotide pool of ADP and ATP which play pivotal role in platelet activation. There is no evidence to show soluble protein cargos in DG lumen. It is suggested that the transporters are involved in their enrichment in DG lumen. Except for the constitutive membrane proteins of DGs, ions play important roles in DG biogenesis and function. Two-pore channel 2 (TPC2) is a component of the DG membrane that regulates the organelle luminal pH and the pool of releasable Ca^2+^ [63]. TPC2 regulates release of Ca^2+^ by ‘kiss-and-run’ events during which two DGs make transient physical contacts and then move away from each other. During these events, DGs exchange contents and may play a role in DG maturation. TPC2 also regulates the formation of membrane tubules connected to DGs [63]. These findings reveal a new mechanism of membrane dynamics in platelet DGs regulated by TPC2.

## Functions of AGs and DGs

Platelet AGs and DGs are both necessary and critical for hemostasis and thrombosis, but the functions of these two granules are different [20,24]. Once the vascular endothelium is injured or in an inflammatory state, platelets form a platelet-rich plug. Platelet function can be considered under the following headings: adhesion, activation, secretion and aggregation [64]. In the process of adhesion, platelets initially bind to collagen exposed by damage to the endothelium via the glycoprotein receptor complex Ib/V/IX expressed on their surface. This process is enhanced by vWF, which is stored and secreted from AGs as well as Weibel–Palade bodies (WPBs) of endothelial cells. When platelets adhere to the damaged vascular endothelium, DGs release a number of stimuli such as ADP to activate platelets. At the same time, platelet activation signaling pathway leads to Ca^2+^ release from DGs. Along with the increasing Ca^2+^ concentration, cAMP concentration decreases and a series of protein kinases such as Src kinase and protein kinase C (PKC) are activated, which in turn induces the release of DG contents, ADP and serotonin, to accelerate the activation and aggregation of platelets to form a hemostatic plug [64].

The deficiencies of AGs and DGs in human genetic disorders manifest with prolonged bleeding, but the phenotypes vary in AG and DG abnormalities. AGs play a pivotal role for normal platelet function as inferred from that ARC syndrome and GPS patients have bleeding diatheses with AG deficiency [65,66]. However, though ARC syndrome and GPS patients have similar phenotypes in AG deficiency, ARC syndrome is more severe than GPS, which seldom survive long because of the loss of essential functions in multiple tissues. GPS is relatively benign which have the primary complications of bleeding, progressive thrombocytopenia and myelofibrosis arising from defective MK development. VPS33B, together with VPS16B, mediates protein sorting and granule maturation that are critical in many tissues, not just in platelets and MKs, while NBEAL2 functions more restricted to MKs and platelets. Perhaps NBEAL2 controls the trafficking of cargo chaperones that are critical for sequestering AG cargos [6]. AGs function widely in hemostasis, thrombosis, and inflammation dependent on the releasing of their contents.

The functions of DGs are independent of AGs as the number of DG is increased in VPS33B-ARC platelets and the absence of VPS16B does not diminish platelet DGs [10,11]. DG biogenesis has been assumed to use similar mechanisms as other LRO, e.g. melanosome. Supporting this idea, several diseases manifest with prolonged bleeding due to DG deficiency together with other manifestations such as OCA, which is caused by defects in melanosomes [7]. For example, HPS patients exhibit bleeding diathesis caused by DG deficiency and hypopigmentation of skin, hair, and eyes due to melanosome defects. Because of HPS gene mutations affect other LRO, some HPS patients present additional phenotypes such as lung fibrosis and immune deficiency [12]. Different HPS subtypes result from mutations in any of ten *HPS* genes in humans, and mutations in at least 15 genes (including orthologs of those ten known *HPS* genes) cause a similar disorder in mice, especially the HPS phenotype in the buff mice with VPS33A mutation [12,15,60,67,68]. In addition, mutations in RAB38 leads to SPD and similar phenotypes of HPS in rat [69]. CHS is caused by mutation of the *CHS1* gene. Due to DG deficiency and multiple defects of other LRO, patients suffering from CHS have bleeding diathesis as well as decreased pigmentation and severe immune deficiency [13]. Mutation of SLC35D3 leads to DG deficiency in platelets or storage pool deficiency (SPD) and metabolic syndrome (MetS) in brain [50,70]. The platelet granule deficiencies and related disorders/genes are summarized in Table 1.

**Table 1:** Platelet granule deficiency and associated diseases/genes

Platelet granule deficiency	Inherited platelet disorder	Genes with mutations
AG deficiency	GPS	*NBEAL2* [9]
	ARC	*VPS33B* [10], *VPS16B* [11]
DG deficiency	HPS	*HPS1 to HPS10* [12,15]
	CHS	*CHS1* [14]
	HPS (mouse)	*VPS33A* [60]
	HPS (rat)	*RAB38* [69]
	SPD (mouse)	*SLC35D3* [50]

## Perspectives

We have learned a lot from platelet granule biogenesis by studying the inherited platelet granule deficiencies [71]. From patients with HPS [72] or CHS [73], the causative genes have been found in the membrane trafficking pathways that affect DG formation. In patients with GPS [65] and ARC [66], mutations of related trafficking genes result in AG defects. Although we have known the defects of AGs or DGs in these inherited disorders, the underlying mechanisms of the defective granules are still very limited. Investigation on AG and DG membrane protein sorting machineries will refine our understanding of the pathways, mechanisms, and molecular machineries involved in different biogenesis of these two organelles and thus better understanding disease pathogenesis. Efforts should be made to find the key proteins in AG or DG biogenesis and the sorting mechanisms for these cargo proteins. Finally, during AG or DG biogenesis, physical contacts with other organelles are required for retrieval or removal of constituents of AGs or DGs. Dissection of these organelle interactions will be helpful to the understanding of platelet granule biogenesis and function.

## Abbreviations

AG: α-granule
AP-3: adaptor protein-3
ARC: arthrogryposis, renal dysfunction, and cholestasis syndrome
BLOC: biogenesis of LRO complex
CHS: Chediak–Higashi syndrome
CORVET: class C core vacuole/endosome tethering complex
DG: δ-granule
FGN: fibrinogen
GPS: gray platelet syndrome
HOPS: homotypic fusion and vacuole protein sorting complex
HPS: Hermansky–Pudlak syndrome
LAMP2: lysosome associated memebrane protein 2
LRO: lysosome-related organelle
MK: megakaryocyte
MRP4: multidrug resistance protein 4
MVB: multivesicular body
MVB I: MVB type I
MVB II: MVB type II
OCA: oculocutaneous albinism
SNARE: soluble NSF attachment protein receptor
SPD: storage pool deficiency
SRC: proto-oncogene c-Src
TGN: *trans*-Golgi network
TPC2: two-pore channel 2
VMAT2: vesicular monoamine transporter 2
VPS33B: vacuolar protein sorting 33 homolog B
vWF: von Willebrand factor
WPB: Weible–Palade body
